# Analysis of antiviral efficacy after switching from brand to generic entecavir in patients with treatment-naïve chronic hepatitis B

This article has been retracted.

**DOI:** 10.1186/s12876-022-02317-7

**Published:** 2022-05-10

**Authors:** Po-Ke Hsu, Pei-Yuan Su, Chia-Lin Wu

**Affiliations:** 1 Division of Gastroenterology, Department of Internal Medicine, Changhua Christian Hospital, Changhua, Taiwan; 2 Institute of Medicine, Chung Shan Medical University, Taichung, Taiwan; 3 School of Medicine, Chung Shan Medical University, Taichung, Taiwan; 4 Division of Nephrology, Changhua Christian Hospital, Changhua, Taiwan; 5 School of Medicine, National Chung Hsing University, Taichung, Taiwan

**Keywords:** Chronic hepatitis B, Generic drugs, Entecavir

## Abstract

**Background/Aims:**

Entecavir (ETV) can suppress chronic hepatitis B (CHB) virus replication as a standard of treatment drugs. For the treatment of CHB, affordable generic drugs may be more widely used in developing and undeveloped countries. However, there is little real-world data regarding the clinical efficacy of switching from entecavir-brand-name drugs (ETV-Brand) to entecavir generic drugs (ETV-Generic) with 0.5 mg once daily. The aim of the study was to evaluate the antiviral activity and safety of ETV-Generic in comparison to ETV-Brand in CHB-patients.

**Methods:**

In this single-center, retrospective, 175 treatment-naïve—CHB-patients were assigned to receive 0.5 mg of ETV-Brand per day for a least 2 years and then switched to ETV-Generic for 6 months for analysis. The primary efficacy endpoint was a sustained virological response in comparison of the rate of undetectable serum Hepatitis B deoxyribonucleic acid (HBV DNA) as the sustained virologic response at baseline and 6 months after switching. Secondary efficacy endpoints were the comparison of the alanine aminotransferase (ALT) levels between before and after switching and ALT normalization. Renal safety consideration was reported on changing the estimated glomerular filtration rate.

**Results:**

From baseline to 6 months, the rate of undetectable HBV DNA and ALT levels remained stable as compared ETV-Brand period with ETV-Generic for 6 months. The rate of undetectable HBV DNA were 81.1%in ETV-Brand versus 88.0%in ETV-Generic (*p* = 0.05 CI 0.1–13.5%). ALT levels were 27.2 IU/L (CI 24.8–29.6 IU/L) in ETV-Brand versus 26.2 IU/L (CI 24.0–28.4 IU/L) in ETV-Generic (*p* = 0.55). Both endpoints were not significantly different between ETV-Brand and ETV-Generic treatments. Kidney function did not significantly differ from ETV-Brand (80.8, interquartile range [IQR]: 66.6–95.3 mL/min/1.73 m^2^) to ETV-Generic treatment period (80.3, IQR: 65.6–93.5 mL/min/1.73 m^2^).

**Conclusion:**

In treatment-naïve CHB-patients, the efficacy and safety profiles of switching from ETV-Brand to ETV-Generic showed no difference. Concluding the ETV-Generic comes to exciting virologic responses and rare adverse events.

**Supplementary Information:**

The online version contains supplementary material available at 10.1186/s12876-022-02317-7.

## Introduction

Hepatitis B is a chronic liver disease caused by hepatitis B virus (HBV) infection, and it is also an important health problem in the world's public health [1]. An estimated 2 billion people worldwide are at risk of HBV, and more than 350 million people are chronically infected [2, 3]. In addition, HBV is also the main cause of liver cirrhosis and hepatocellular carcinoma (HCC). Therefore, controlling HBV to prevent liver cancer and cirrhosis has become a very important issue [4]. The global HBV infection rate varies by geographic region, and the prevalence of healthy carriers ranges from 0.1 to 15% [5, 6]. In Taiwan, with the implementation of the Viral Hepatitis Control Program (VHCP) in the 1970s and the launch of the universal vaccination program in 1984, the HBV infection rate among the general population dropped significantly from 15–20 to 1% [7–11].

The standard of chronic hepatitis B (CHB) treatment is to suppress the amount of HBV virus. By inhibiting the quantity and activity of HBV, it reduces inflammation and prevents fibrosis, liver cirrhosis, liver failure and even HCC. Thereby, it is possible to reduce mortality due to liver disease and to improve the survival rate. The treatment goal is loss of hepatitis B surface antigen (HBsAg), but complete eradication of HBV is nearly impossible, because nuclear covalently closed circular DNA (cccDNA) remains in the liver cell [12, 13]. In clinical practice, normalization of alanine aminotransferase (ALT), undetectable serum HBV DNA, and improvement of histological inflammation or fibrosis are indicators of treatment response [14].

Entecavir (ETV) is a deoxyguanosine nucleoside analog which exerts antiviral effects by inhibiting three steps of replication: priming of HBV DNA polymerase, reverse transcription of the HBV DNA negative strand from pregenomic mRNA, and synthesis of the HBV DNA positive strand [15]. Generic ETV (ETV-Generic) had been introduced to the market since 2019 in Taiwan and with an advantage of a lower price that more CHB-patients can be treated.

Envir® is a generic ETV drug developed by China Chemical & Pharmaceutical (CCPC) equivalent in laboratory tests to the brand-name ETV drug (Baraclude®, ETV-Brand) by Bristol-Myers Squibb (BMS). Previous studies similar antiviral efficacy with regard to switching from brand-name to generic ETV 1 mg for antiviral-resistant chronic hepatitis B [16, 17]. Due to the influence of Taiwan's insurance policy, the utilization rate of Generic ETV (ETV-Generic) has greatly increased in recent years. However, there is a lack of real-world data evaluating the efficacy and safety of switching from brand-name to generic ETV 0.5 mg for controlling CHB. Therefore, the current study was designed to compare the antiviral efficacy and safety between lower dose brand-name and generic ETV in CHB-patients.

## Materials and methods

### Study design

This study was conducted using a single-center retrospective real-world medical database in Changhua Christian Hospital from January 1, 1999, to December 31, 2019. All patients were treated or followed in the hospital. In December 2018, stable CHB-patients under the treatment of 0.5 mg ETV-Brand were informed to switch the treatment to 0.5 mg ETV-Generic. All the informed consents of the participants were given before changing their treatment. Then their treatment was changed for 1 year (from January 1, 2019, to December 31, 2019). After switching for 1 year, our retrospective study compared patient efficacy and safety using hospital medical databases. The study was carried out in compliance with the declaration of Helsinki and was approved by the Institutional Review Board of Changhua Christian Hospital (approval number: 210202). The study was performed in compliance with good clinical practices, according to the International Conference on Harmonization (ICH) guidelines.

### Patient enrollment

Inclusion criteria were male and female patients of ages 18–75 years who were diagnosed as HBsAg-positive since January 1, 1999, to December 31, 2019 and had a medical record of CHB under the ETV-Brand for 2 years. No other anti-viral medications during the study period of time were recorded. Exclusion criteria included: (1) Age < 18 years; (2) Transfer to other hospital; (3) Virologic resistance to ETV-Brand; (4) Switching to Tenofovir; (5) Switching time less than 48 weeks (without enough observation time). Finally, 175 patients were eligible for the analysis of effectiveness and renal safety (Fig. 1).

**Fig. 1:** Study flowchart. ETV-Brand, entecavir-brand drugs; NAs, nucleoside analogues; IFN, interferon; ETV-Generic, entecavir-generic drugs; ALT normalization, alanine aminotransferase normalization; SVR, sustained virological response

## Study outcome

### Sustained virologic response and alanine aminotransferase (ALT) stabilization

The primary endpoint was evaluated by sustained virologic response rate defined by undetectable HBV DNA which means HBV DNA viral load < 10 IU/mL between baseline (on 0.5 mg ETV-Brand for at least 6 months) and after switching to 0.5 mg ETV-Generic for 6 months. The secondary endpoint was evaluated by comparing the serum ALT levels before and after switching (ALT normalization).

### Renal safety

Comparison of renal safety of ETV-Brand and ETV-Generic was defined as the renal function (eGFR) before switching and after switching for 6 months.

### Statistical analysis

All efficacy analyses were performed on the full analysis set. The population included all analytical subjects who received at least once daily dose of ETV-Brand for 2 years as baseline characteristics. For sample size calculation, a one-sided α level of 0.025 and 80% power, a sample size of 102 patients was estimated with a noninferiority margin of one. Considering a 20% drop-out rate, the study will require a total of 126 patients.

For the primary efficacy of sustained virologic response rateand secondary efficacy of ALT level change, we use paired *t*-test for comparing the two treatment modalities. Change in renal function (eGFR) between the two treatment modalities was also analyzed by using paired *t*-test. All statistical analyses were performed using SAS version 9.4 (SAS Institute Inc., Cary, NC, USA) and MedCalc® Statistical Software version 20.008 (MedCalc Software Ltd, Ostend, Belgium; https://www.medcalc.org; 2021).

## Results

### Baseline characteristics

The median age of the included patients was 61 (IQR: 52.5–68.8) years, and male sex was predominant (68.0%). The median treatment period of CHB with ETV was 3.2(IQR: 2.7–4.3) years, and all patients were treatment-naïve. The rate of HBeAg positivity was 19.4%. And the median Fibrosis-4 (FIB-4) Index for Liver Fibrosis was 2.7 (IQR: 2.2–3.0). Mean detectable HBV DNA level showed 14.0 (12.4–16.5) IU/mL, see Table 1.

**Table 1:** Baseline characteristics of the patients included in study group

Characteristic	Initial treatment of ETV-Brand
Age, years	61 (52.5–68.8)
Male sex, n (%)	119/175 (68.0%)
BMI, kg/m^2^	24.3 (22.2–27)
Period of ETV-Brand(years)	3.2 (2.7–4.3)
WBC, × 10^3^/μL	5.8 (4.4–7.3)
HB, g/dL	13.8 (12.7–14.6)
Platelet, × 10^3^/μL	145 (104–191)
ALT, U/L	24 (18–32)
AST, U/L	29 (24–36)
Total bilirubin, mg/dL	0.8 (0.6–1.1)
eGFR, mL/min/1.73 m^2^	81.8 (78.8–87.2)
FIB-4 score	2.7 (2.2–3.0)
HBeAg-positive, n (%)	34 (19.4%)
Detectable HBV DNA level, IU/mL	14.0 (12.4–16.5)
Undetectable HBV DNA, n (%)	142/175 (81%)

Data are expressed as n (%) for categorical data and as mean ± standard deviation or median (interquartile range) for continuous data

ETV-Brand, entecavir-brand drugs; BMI, body mass index; WBC, white blood cell; HB, hemoglobin; ALT, alanine aminotransferase; AST, aspartate aminotransferase; eGFR, estimated glomerular filtration rate; FIB-4, Fibrosis-4; HBeAg, Hepatitis B e antigen; HBV DNA, hepatitis B virus deoxyribonucleic acid

### Primary end point of efficacy: comparison of sustained virologic response rate between initial baseline data and 6 months data of the treatment of ETV-Generic

After 2 years treatment of ETV-Brand as the proportion of patients with undetectable HBV DNA and comparing of 6 months treatment of ETV-Generic, it showed 142 (81%) to 154 (88%) without significant, *p* = 0.05, see Fig. 2.

**Fig. 2:** Comparison of undetectable HBV DNA between initial baseline data and 6 months data of the treatment of ETV-Generic reported no significant, *p* = 0.05, showing the anti-viral efficacy maintained. HBV DNA, Hepatitis B deoxyribonucleic acid; ETV-Brand, entecavir-brand drugs; ETV-Generic, entecavir-generic drugs

### Secondary end point of efficacy: comparing initial ALT and 6 months data of the treatment of ETV-Generic

For all included patients, ALT kept normal from Brand to Generic with ALT: 27.2 IU/mL (CI: 24.8–29.6) to 26.2 IU/ml (CI 24.0–28.4) respectively showed no significant, *p* = 0.55, see Fig. 3.

**Fig. 3:** Comparison of ALT between initial and the 6th month data of the treatment of ETV-Generic reported no significant, *p* = 0.55, showing sustained ALT normalization. ALT, alanine aminotransferase; ETV-Brand, entecavir-brand drugs; ETV-Generic, entecavir-generic drugs

### Adverse events

All adverse events were recorded showed no significant symptoms during the treatment either ETV-Brand or ETV-Generic. The major safety profile was a renal outcome issue of eGFR changes. Comparing with ETV-Brand and ETV-Generic, eGFR changes showed 80.8 mL/min/1.73 m^2^ (IQR: 66.6–95.3) to 80.3 mL/min/1.73 m^2^ (IQR: 65.6–93.5) without statistical significant, *p* = 0.59, see Fig. 4.

**Fig. 4:** Comparing with ETV-Brand and ETV-Generic, eGFR changes showed no statistical significance, *p* = 0.59. Suggesting the switching from ETV-Brand to ETV-Generic is safe. eGFR, estimated glomerular filtration rate; ETV-Brand, entecavir-brand drugs; ETV-Generic, entecavir-generic drugs

## Discussions

In this real-world study, we found the switching from ETV-Brand to ETV-Generic is safe and the anti-viral efficacy was maintained.

CHB imposes a significant global health care burden; approximately 5% of individuals throughout the world are estimated to be infected with HBV [18], and the annual mortality associated with persistent HBV infection is more than 1 million per year [19]. Mother-to-child transmission is the driving force of new HBV infections in high prevalence countries especially in Asia [20, 21].

In addition to making national wide-ranging treatments possible through standard therapies, affordable entecavir will benefit more HBV patients. With the popularization of hepatitis B vaccination, significant effects have been achieved in suppressing the spread of hepatitis B virus [22]. Therefore, by treating more than 350 million chronically infected people, the continued spread of the virus can be prevented [23]. International guidelines recommend ETV and tenofovir (TDF) as the first-line therapy for initial CHB-patients because of its strong antiviral activity and higher genetic barrier [24, 25]. Compared with TDF, basic patents expire in 2017 [26], entecavir is already generic in several countries, including the United States of America (USA) and Europe. In 2017, due to the introduction of tenofovir and entecavir generics in Germany, the treatment costs decreased by 31% with average therapy costs at 498 Euro per patient per month in 2016 and decreased to 214 Euro in 2019 and causing the increase the number of CHB-patients on treatment leading to the prevention of progression to more severe disease [27]. The basic patent for ETV-Brand in the USA was invalidated in 2014 [28]. In China and Brazil, the basic patents expired in 2011 [29]. In terms of price, generic ETV can be more feasible in developing or undeveloped country [30].

Generic medication is common in use for hypertension such as Amlodipine Besylate (Norvasc®) after the patent invalidated in 2007. Previous studies had shown the same efficacy comparing with generic and brand medication [31]. For now, there is little data regarding the real-world result of efficacy of using generic anti-viral therapy in chronic hepatitis B.

We acknowledge that there are several limitations, including small sample size and no placebo control study, retrospective not randomized study, and a single center study. Further studies with a prospective, quasi-experimental approach still highly needed to explain the further effectiveness and safety of ETV-Generic.

The advantages of this study are (1) A first real-world data comparing ETV-Brand to ETV-Generic in Asian countries (2) Pointing out of generic drugs for virus eradication especially of CHB in the global health is important.

## Conclusion

In patients with previously untreated HBV infection, the efficacy and safety profiles of switching from ETV-Brand to ETV-Generic showed no difference. Concluding the ETV-Generic comes to exciting virologic responses and rare adverse events. Therefore, affordable generic drugs may be widely used in undeveloped and developing countries to treat hepatitis B. But it still needs to be confirmed by further studies in the future.

## Supplementary Information

**Additional file 1:** Raw data.

## Data Availability

All data generated during this study are included in this published article and Additional file 1 of Raw data.
